RETRACTED

# Construction of a Prediction Model for College Students' Psychological Disorders Based on Decision Systems and Improved Neural Networks

**DOI:** 10.1155/2022/6746419

**Published:** 2022-07-05

**Authors:** Ming Li, Jiming Feng

**Affiliations:** Northeast Petroleum University, Daqing, Heilongjiang 163318, China

## Abstract

Modeling and prediction of psychological disorders is a hot topic in current research. Neural networks are very important factors in improving the accuracy and precision ratios of the models which are developed for the prediction of the psychological disorders. An upgraded neural network prediction model of psychological diseases was suggested in order to attain an optimum prediction effect of psychological disorders. First, it analyzes the current progress in predicting the psychological barrier, finds the current limitations of various psychological barrier forecast model, collects the historical data of psychological barriers, and introduces the chaos algorithm of mental disorder history data preprocessing, psychological barriers to better mining change characteristic, and then, after pretreatment using neural network to the psychological barriers to learning history data, introduce the grain subgroup algorithm to improve the problems existing in the neural network, establish a prediction model of the optimal psychological barriers, and finally, through the contrast test and other psychological obstacle prediction model, the results depict enhanced neural network psychological barrier prediction accuracy of more than 95%, compared with the contrast model. Precision is improved by more than 5%. At the same time, the psychological barrier modeling time is shorter, improving the psychological barriers to predict. The efficiency has a higher practical application value.

## 1. Introduction

As people's living pressure rise, a segment of the population may develop a psychological disease; mental disorder is a common mental disease; mild mental disorders can be treated with self-regulation; and serious psychological barrier problems require treatment; thus, psychological barrier problems have emerged as a significant problem in people's lives. The occurrence of psychological barriers is a long process of accumulation, and forecasting the degree of psychological barrier to development can help people understand the psychological barriers in advance, as early as possible, to make some adjustments and treatment measures with a low probability of occurrence of psychological barriers. Thus, the psychological barrier prediction research becomes the psychological direction of a hot spot in data mining.

Due to the increasing pressure in society, family, and life, many people have psychological disorders of varying degrees. Psychological disorders have certain negative effects on numerous aspects such as harmony, happiness, and social stability of the family [1–3]. Prediction and modeling of psychiatric diseases can aid relevant authorities and researchers in better understanding the features of these disorders. As a result, psychological disorder prognosis has a significant societal and practical significance [4–6].

RETRACTED

Initially, some experts were used to predict psychological sicknesses. Prediction results of psychological disorders by this method were unstable, and different experts could get different results. And, the prediction results are closely related to the experts' own knowledge richness, which makes the prediction results of psychological disorders quite subjective and the reliability of the prediction results of psychological disorders low [7, 8]. Then, the Bayes inference prediction model of psychological disorders based on the analytic hierarchy process (AHP) emerged, in which AHP is a linear modeling method. And, psychological barriers with time-varying change, namely, the so-called nonlinear, make it unable to fully describe the psychological barrier change point. The psychological barrier forecast error is large, and there is also a psychological barrier forecast model based on the Bayes reasoning the low accuracy of shortcomings.

In the last ten years, people have continued to explore the subject of psychological disorder prediction in depth and have produced several promising discoveries as well as numerous useful psychological disorder prediction models. The conventional psychological disorder prediction model and the current psychological disorder prediction model are the two types of psychological disorder prediction models. Traditional psychological barrier forecast model with traditional mathematical modeling methods, such as multiple linear regression and analysis of mental disorder history data, find the corresponding coefficient of multiple linear regression, establish the corresponding psychological obstacle forecast model, and forecast the psychological barrier of simplified to the psychological barrier problem for a period of time in the future estimates.

Artificial neural network by simulating human brain works to automatic solving problems, in particular, the BP neural network has been widely used in many fields [9]. The modeling effect of the BP neural network is closely related to the selection of initial connection weights and thresholds. If the selection is not reasonable, the neural network cannot effectively converge in the training process and is prone to fall into local extreme values [10, 11]. In order to improve the prediction accuracy of mental disorders, this paper puts forward an improved neural network prediction model of mental disorders and verifies the superiority of the improved neural network through simulation experiments. This model has the capacity to improve the accuracy of the underlined model with an exceptional ratio.

RETRACTED

The rest of the paper is arranged according to the following criteria.

In Section 2, a description of the improved neural network prediction model is presented, wherein, initially, the back propagation neural network is defined. Results of the experiments or simulations are presented in Section 3 following the prediction model. Lastly, we have presented a summary of the work.

## 2. Improved Neural Network Prediction Model

A neural network (NN) is a machine learning (ML) approach for training computers to analyse data by mimicking the brain of a human being. Deep learning is a particular branch of machine learning which is based on the idea of nodes or neurons (preferably connected) in the form of layers that is quiet like the brain of a human. Each connection, like the human brain's synapses, may transmit an indication to the neighboring neurons. A neuron (artificial here) collects and evaluates electrical impulses prior to sending messages to the neighbors neurons. A nonlinear procedure of a neuron's inputs determines its output, and the “signal” at a connection is a real number. Edges are the terms used to describe connections. The weight of neurons and edges is frequently changed as learning progresses.

### 2.1. BP Neural Network

Backpropagation denotes the process which is used for the gradient computation, no concern about its utilization; nonetheless, BP is sometimes used loosely to point to the expected learning process, particularly complete, which surely includes information about the usage of the gradient, that is, similar to the stochastic gradient descent. The BP neural network is a multiple layered feedforward network with error back propagation that can match nonlinear high-precision input and output relations without understanding the problem's mathematical representation. It is made up of three layers: input, concealed, and output.  Figure 1 depicts a description of the fundamental structure [12].

Let the training set be (*X*^*k*^, *Y*^*k*^), *k*=1,2,…, where *X*^*k*^ and *Y*^*k*^ represent the input and output of the *k*-th sample, respectively. Specifically, *X*^*k*^=(*x*_1_^*k*^, *x*_2_^*k*^,…, *x*_*n*_^*k*^) and *Y*^*k*^=(*y*_1_^*k*^, *y*_2_^*k*^,…, *y*_*n*_^*k*^) correspond to the corresponding neuron nodes. If the output of the neural network is consistent with the expected value, the learning process of the BP neural network will be terminated; otherwise, the error between the two will be calculated, and the connection weight and threshold will be adjusted according to the error until the output of the neural network is consistent with the expected value. The connection weights between the *i*^th^ and *h* nodes of hidden and input layers and the *j*-th node of the output layer are *w*_*hi*_^1^  and *w*_*ij*_^2^, respectively. For the *j*-th node of the output layer, the error calculation formula of the KTH sample on the output layer is

(1) $$\begin{array}{c} E_{k}=\frac{1}{2}\overset{m}{\underset{j=1}{\sum }}{\left(y_{j}-y_{j}^{k}\right)}^{2},\;k=1,2,\ldots ,q. \end{array}$$

For the entire training sample set, the formula for calculating the overall error is

(2) $$\begin{array}{c} E=\overset{q}{\underset{k=1}{\sum }}E_{k}. \end{array}$$

For the *j*-th node in the output layer, its weighted input and actual output are, respectively,

(3) $$\begin{array}{c} {\text{nety}}_{j}=\overset{p}{\underset{i=1}{\sum }}\left(b_{i}{}^{*}w_{ij}^{2}-\theta_{j}\right), \end{array}$$

(4) $$\begin{array}{c} y_{j}=f\left(\text{net}y_{j}\right). \end{array}$$

In the equation, *θ*_*j*_ represents the threshold value of the hidden layer; *p* represents the node of the hidden layer; and *f* (*x*) represents the activation function of the node, as follows:

(5) $$\begin{array}{c} f\left(u\right)=\frac{1}{1+{\text{e}}^{-u}}. \end{array}$$

The weighted input and actual output of the hidden layer node *I* connected to the output layer node *J* are shown in

(6) $$\begin{array}{c} {\text{netb}}_{i}=\sum^{}\left(x_{h}*w_{hi}^{1}-\theta_{i}\right), \end{array}$$

(7) $$\begin{array}{c} b_{i}=f\left(\text{net}b_{i}\right). \end{array}$$

In the equation, *θ*_*i*_ represents the threshold for the output layer. Since *f* (*u*) is a function that can decrease slightly, the generalized error of node *J* at the output layer can be expressed as

(8) $$\begin{array}{c} d_{j}=-\frac{\partial E_{k}}{\partial \text{net}y_{i}}. \end{array}$$

Formula (9) can be obtained by combining formulas (3) and (8).

(9) $$\begin{array}{c} d_{j}=-\frac{\partial E_{k}}{\partial y_{j}}\frac{\partial y_{j}}{\partial \text{net}y_{j}}=-\frac{\partial E_{k}}{\partial y_{j}}f^{\text{'}}\left(\text{net}y_{j}\right). \end{array}$$

By combining equations (1) and (10), the following can be obtained:

(10) $$\begin{array}{c} \frac{\partial E_{k}}{\partial y_{j}}=\frac{\partial \left[\left(1/2\right)\sum_{j=1}^{m}{\left(y_{j}-y_{j}^{k}\right)}^{2}\right]}{\partial y_{j}}. \end{array}$$

According to the function property of weak decreasing *f*(), the following can be obtained.

(11) $$\begin{array}{c} f\left(\text{net}y_{j}\right)=y_{j}\left(1-y_{j}\right). \end{array}$$

Synthesis formula (9): formula (11) produces

(12) $$\begin{array}{c} d_{j}=y_{j}\left(1-y_{j}\right)\left(y_{j}^{k}-y_{j}\right). \end{array}$$

The generalization error of node *I* of the hidden layer can be expressed as

(13) $$\begin{array}{c} \Delta e_{i}\Delta =-\frac{\partial E_{k}}{\partial \text{net}b_{i}}=-\frac{\partial E_{k}}{\partial b_{i}}\frac{\partial b_{i}}{\partial \text{net}b_{i}}=-\frac{\partial E_{k}}{\partial b_{i}}f^{\text{'}}\left(\text{net}b_{i}\right)\Delta \Delta =-\overset{m}{\underset{j=1}{\sum }}\left(\frac{\partial E_{k}}{\partial \text{net}y_{j}}\frac{\partial \;net\;y_{i}}{\partial b_{i}}f^{\text{'}}\left(\text{net}b_{i}\right)\right). \end{array}$$

Equation (14) can be obtained by combining equations (8) and (3).

(14) $$\begin{array}{c} \Delta e_{i}\Delta =\overset{m}{\underset{j=1}{\sum }}d_{j}\frac{\partial \left[\sum_{i=1}^{p}b_{i}*w_{ij}^{2}\right]}{\partial b_{i}}f^{\text{'}}\left(\text{net }b_{i}\right)\Delta \Delta =\overset{m}{\underset{j=1}{\sum }}d_{j}*w_{ij}^{2}*f^{\text{'}}\left(\text{net }b_{i}\right). \end{array}$$

Similar to formula (11), the following can be obtained:

(15) $$\begin{array}{c} f\left(\text{net }b_{i}\right)=b_{i}\left(1-b_{i}\right). \end{array}$$

Then, equation (14) becomes

(16) $$\begin{array}{c} e_{i}=b_{i}\left(1-b_{i}\right)\sum_{j=1}^{m}d_{j}*w_{ij}^{2}. \end{array}$$

The gradient descent algorithm is adopted to reduce the overall error *E*_*k*_. Since there is a proportional relationship between the connection weight and (−*∂E*_*k*_/*∂w*_*ij*_^2^), the variation forms of *w*_*hi*_^1^ and *w*_*ij*_^*i*^ are

(17) $$\begin{array}{c} \Delta w_{ij}^{2}=-\alpha \frac{\partial E_{k}}{\partial \text{ net }y_{j}}\frac{\partial \text{ net }y_{j}}{\partial w_{ij}^{2}}=\alpha d_{j}\left[\frac{\partial \left(\sum_{i=1}^{p}b_{i}w_{ij}^{2}\right)}{\partial w_{ij}^{2}}\right], \end{array}$$

(18) $$\begin{array}{c} \Delta w_{ij}^{1}=-\beta \frac{\partial E_{k}}{\partial w_{ij}^{1}}=-\beta \frac{\partial E_{k}}{\partial \text{ net }b_{i}}\frac{\partial_{net}b_{i}}{\partial w_{ij}^{1}}=\beta e_{i}x_{h}, \end{array}$$

where *α* and *β* are the learning rate. In order to improve the convergence speed of the neural network, the momentum increasing term is introduced, and the following equations are obtained:

(19) $$\begin{array}{c} \Delta \Delta w_{ji}^{r}\left(s+1\right)=\Delta \eta \frac{\partial E}{\partial w_{ji}^{r}}+\rho \Delta w_{ji}^{r}\left(s\right)\Delta \Delta \left(0<\rho <1\right),\;r=1,2, \end{array}$$

(20) $$\begin{array}{c} \Delta w_{ji}^{r}\left(s+1\right)=w_{ji}^{r}\left(s\right)+\Delta w_{ji}^{r}\left(s+1\right),\;r=1,2, \end{array}$$

where *S* represents the number of iterations.

RETRACTED

The prediction and modeling effect of psychological disorders of the BP neural network is closely related to the selection of initial connection weights and thresholds. If the selection is not reasonable, the neural network cannot effectively converge in the training process and is easy to fall into local extreme values. Therefore, the PSO algorithm is selected in this paper to determine the initial value of connection weights and thresholds.

### 2.2. Particle Swarm Optimization Algorithm

In computational science, PSO is a computer technique for optimising an issue through a repeated attempt so that the probability of the candidate solution is increased in terms of a given quality metric. There are *n* particles in a d-dimensional space, which form a set *X* = (*X*_1_,*X*_2_,…, *X*_*n*_). The position and velocity vector of the *i*th particle are, respectively, *X*_*i*_ = (*x*_i1_,*x*_i2_,…, *x*_*iD*_) and *V*_*i*_=(*v*_*i*1_, *v*_*i*2_,…, *v*_*i*  *D*_). The first particle quality evaluation is realised by the fitness function, and individuals and particle swarm are in the best position in historical information.

(21) $$\begin{array}{c} v_{ij}^{k+1}=\omega v_{ij}^{k}+c_{1}r_{1}\left(P_{ij}^{k}-x_{ij}^{k}\right)+c_{2}r_{2}\left(P_{gj}^{k}-x_{ij}^{k}\right), \end{array}$$

(22) $$\begin{array}{c} x_{ij}^{k+1}=xv_{ij}^{k}+v_{ij}^{k+1}, \end{array}$$

where *k* represents the number of iterations; *c*_1_ and *c*_2_ represent acceleration factors; and *ω* is inertial weight.

In the PSO algorithm, the acceleration factor and inertia weight are fixed, and the individual diversity of the particle swarm will gradually weaken with the increase of the iterations number and also gradually enter the local optimal solution. Therefore, the standard PSO algorithm is improved in this paper as follows:

(23) $$\begin{array}{c} \;\left\{\begin{array}{c} \Delta \Delta \omega^{k}=\left[\left(\omega_{0}-\omega_{1}\right)\cos\left(\frac{\pi k}{K}\right)+\frac{\left(\omega_{0}+\omega_{1}\right)}{2}\right],\\ \Delta \Delta c_{1}^{k}=c_{10}-\left(c_{10}-c_{11}\right)\left(\frac{1-k}{K}\right),\\ \Delta \Delta c_{2}^{k}=c_{20}+\left(c_{21}-c_{20}\right)\left(\frac{1-k}{K}\right). \end{array}\right) \end{array}$$

### 2.3. Improved Neural Network Prediction Model Design of Psychological Disorders

Distressing, debilitating and/or aberrant thoughts, feelings, and behaviours are all symptoms of a psychiatric condition. Psychopathology is the scientific study of psychiatric disorders, including their symptoms, aetiology (causes), and treatment. To improve psychological barriers of neural network prediction model of working principle, first, we collect the historical data of psychological disorders, and then use chaos algorithm to preprocess the historical data of psychological disorders, which will better mine the changing characteristics of psychological disorders. Finally, after preprocessing, we use neural network to learn the historical data of psychological disorders, and use particle swarm optimization algorithm to solve the optimization problem of neural network. The optimal prediction model of psychological disorders was established as shown in Figure 2.

RETRACTED

The steps of improving neural network to predict psychological disorders are as follows:

Step l: the historical number of mental disorders is used in this study to determine the prevalence of mental diseases. They construct a time series data based on the data without taking into account the important influencing elements, resulting in a one-dimensional time series data.
Step 2: since the historical data is a one-dimensional time series data, the BP neural network cannot be trained. Combined with the time variability of psychological obstacle changes, the chaos algorithm is introduced to transform one-dimensional time series data into multidimensional time series data by introducing embedding number (*M*) and time delay (*z*), that is, embedding number represents the heart of the current time point! The prevalence of psychological disorders was correlated with the previous prevalence data of several psychological disorders. The time delay represented the interval between data points, and the data were divided into training sets and tests.
Step 3: initialize the BP neural network and determine the number of nodes in the input layer of the BP neural network according to the embedding number (*m*). The output layer is the predicted value of psychological disorder, that is, one. Nodes that belong to the hidden layer are actually in input layer (*m*) multiply by 2 plus 1, i.e., 2*m* + 1.
Step 4: construct the fitness function of the PSO algorithm. In this paper, the prediction of psychological disorders is taken as the fitness function, which can be expressed as
  (24) $$\begin{array}{c} F=\sum_{j=1}^{m}{\left(y_{j}-y_{j}^{k}\right)}^{2}. \end{array}$$
Step 5: according to the *i*-th and *h* nodes of hidden and input layers, respectively, the initial connection weights *w*_*hi*_^1^ and *w*_*ij*_^*i*^ between the point and the *j*-th node of the output layer, and the initial threshold of the hidden layer and the output layer is *θ*_*i*_ and *θ*_*j*_ and initialize the position of the particle.
Step 6: calculate the fitness function of each particle and determine the optimal location of the individual and particle swarm in the first iteration.
Step 7: update the particle position and velocity according to equations (21) and (22).
Step 8: the number of iterations is increased until the optimal particle position is found, and the initial connection weight and threshold are obtained according to the optimal particle position.
Step 9: BP neural network obtains the initial connection weight according to the optimal particle position and threshold to learn the training sample set of psychological disorders and establish the optimal psychological disorders prediction model.
Step 10: test and verify the performance of the test sample psychological disorder prediction model.

RETRACTED

## 3. Simulation Results

In order to validate the proposed scheme, extensive simulations were carried out in MATLAB, and various results are presented along with both textual and graphical explanations. Moreover, these results, those of the proposed schemes, are matched with the existing field proven approaches. For simplicity, it is divided into various sections such as data and the environment.

### 3.1. Experimental Environment and Data

In order to analyse and improve the performance of neural network's psychological disorder prediction model, a simulation experiment was conducted, and the experimental environment is shown in Table 1.

In order to make the experimental results of the improved neural network comparable, the standard BP neural network (BPNN) and the standard PSO algorithm (PSO-BPNN) were selected to optimize the BP neural network for the comparison experiment of mental disorders prediction. A total of 500 historical data of mental disorders were collected. Chaos algorithm was used to determine the embedding number *M* = 5 and time delay = 4, with different choices. Five simulation experiments of psychological disorder prediction were performed on the training samples.

### 3.2. Experimental Results and Analysis

The parameters of PSO are set as follows: population size is 10; the maximum number of iterations is 200; and the value range of *c* is [2,3]. The value range of C2 is [0.5, 2]. The value range of *c* is [0.5,1]. And, the BP neural network is 0.1. Three models are used to learn the mental obstacle training samples in Table 2, and then the test samples are predicted, and the prediction accuracy of their mental obstacle is counted. The results are shown in Figure 3.

It can be known from the analysis of Figure 3 [1]. The prediction accuracy of the standard BP neural network for psychological disorders is the lowest, which is below 85%, making the prediction of psychological disorders over 15%, which cannot meet the practical application requirements of psychological disorders prediction [2]. The prediction accuracy of psychological disorders optimized by the standard PSO BP neural network is higher than that of the standard BP neural network, indicating that introducing the PSO algorithm to optimize the connection weight and threshold value of BP neural network is beneficial to improve the prediction effect of psychological disorders. [3] Compared with the standard BP neural network and standard PSO algorithm. In this paper, the BP neural network prediction model of psychological disorders is established. The accuracy of the model established in this paper is higher than that of the BP neural network optimized by the standard particle swarm optimization algorithm by more than 5%. While optimizing the connection weight and threshold of the BP neural network, the particle swarm optimization algorithm is correspondingly improved to obtain a more ideal prediction of psychological disorders. The difficulty of network in the modeling of mental disorder prediction greatly reduces the error of mental disorder prediction and has obvious advantages.

RETRACTED

The mental obstacle training time and test time of different models were counted, and the results are shown in Figure 4.

Comparing the training time and testing time of psychological disorders in Figure 4, it can be found that the training time and testing time of the standard BP neural network of psychological disorders are the longest. This paper uses the standard particle swarm optimization algorithm to optimize the BP neural network. It can also be seen from Figure 4 that the model time of this paper is the shortest. It shows that, in the process of modeling in this paper, the BP neural network speeds up the convergence speed and reduces the idea to get the optimal BP neural network. This is mainly because the improved PSO algorithm obtained better connection weights and thresholds, which improved the modeling efficiency of mental disorders prediction.

## 4. Conclusion

A mental disorder prediction model based on upgraded neural networks is developed in order to get the structure of mental illness prediction with greater accuracy. The findings demonstrate that the enhanced neural network solves the shortcomings of the present mental disease prediction model, and that it is a mental disorder prediction model with high accuracy and efficiency and a broad range of applications.

Effective strategies of health education and health promotion for persons with mental disorders are as follows: (1) strengthen the publicity of mental health and enhance the social attention to mental health including physical health and mental health in three parts. There are still some people's understanding of health which only stays at the level of “physical health,” ignoring the attention and protection of their own and their relatives' mental health. (2) We should actively carry out the inspection and screening of mental disorders. In promoting the health education and health work of patients with mental disorders, the state and the government should also actively carry out the self-examination and screening of mental disorders so as to help people from all walks of life face the problem of mental disorders and achieve early detection and early treatment. (3) Patiently listen to the appeal of patients with psychological disorders and psychological counseling in the diagnosis of mental disorders of patients with health education and health promotion work, should be patient to listen to the appeal of patients with psychological disorders, and timely give psychological counseling, help patients to stabilize the state of mind, calm in the face of difficulties, and alleviate psychological abnormalities. When listening, patients with psychological disorders should be fully respected, patients' privacy should be protected, patients' extreme thinking and behavior should be corrected, and a good mental health care environment should be created to promote patients' rehabilitation.

RETRACTED

## Figures and Tables

**Figure 1:** General architecture of the BP neural network.

**Figure 2:** The working principle of the neural network prediction model of mental disorder was improved.

**Figure 3:** Comparison of prediction accuracy of psychological disorders in different models.

**Figure 4:** Comparison of modeling efficiency of different models for predicting psychological disorders.

**Table 1:** Simulation experiment environment setting.

Parameter names	The parameter value
CPU	4 core Intel
RAM	32 GB
OS	WIN 10
Programming tools	MATLAB 2019

**Table 2:** Sample distribution of simulation training and test for psychological disorder prediction.

The serial number	The parameter value
1	1 : 1
2	2 : 1
3	3 : 1
4	4 : 1
5	5 : 1

## Data Availability

The data used to support the findings of this study are available from the corresponding author upon request.
